# Effect of Wrist Dorsiflexion/Palmar Flexion on Median Nerve Deviation and Cross-Sectional Area in Patients with Carpal Tunnel Syndrome

**DOI:** 10.1155/2023/3631193

**Published:** 2023-02-01

**Authors:** Lei Xu, Tao Ma, Min Zhang, Linjie Zhou, Caizhi Hu

**Affiliations:** Department of Hand and Foot Surgery, Yijishan Hospital of Wannan Medical College, Wuhu, Anhui, 241000, China

## Abstract

**Objective:**

To evaluate the effect of wrist dorsiflexion/palmar flexion on median nerve excursion and cross-sectional area in patients with carpal tunnel syndrome.

**Methods:**

From November 2019 to December 2021, 85 patients (110 affected wrists) who presented to our department and were diagnosed with carpal tunnel syndrome were collected and classified by severity as mild to moderate. Twenty-five healthy controls were selected during the same period, with a total of 50 healthy wrists. All patients and healthy volunteers underwent high-frequency ultrasonography to measure the vertical deviation between the median nerve and the transverse carpal ligament during wrist dorsiflexion/palmar flexion and the changes in the cross-sectional area of the median nerve in the pisiform plane. All patients with carpal tunnel syndrome underwent neurophysiological testing to measure median nerve sensory conduction velocity, sensory latency time, and sensorimotor point fluctuation amplitude.

**Results:**

The mean age of the patients was 50 ± 8 years, the proportion of males was 18%, and the disease course was 2.3 ± 1.2 years. In terms of severity grading, 38 patients (34.5%) had mild carpal tunnel syndrome, 30 patients (27.3%) had moderate carpal tunnel syndrome, and 42 patients (38.2%) had severe carpal tunnel syndrome. Compared with the control group, the distance between the proximal median nerve and the transverse carpal ligament, the distance between the distal median nerve and the transverse carpal ligament, and the cross-sectional area were decreased in the carpal tunnel syndrome group compared with those during wrist dorsiflexion, and the differences were statistically significant (*P* < 0.05). Compared with the control group, there were significant differences in the vertical distance and cross-sectional area between the median nerve and the transverse carpal ligament at the proximal and distal ends in the mild, moderate, and severe groups (*P* < 0.05). The proximal vertical distance of the median nerve was positively correlated with sensory latency (*P* < 0.05) and negatively correlated with sensory conduction velocity (*P* < 0.05). The vertical distance of the distal end of the median nerve was also significantly positively correlated with sensory latency (*P* < 0.05) and significantly negatively correlated with sensory conduction velocity (*P* < 0.05).

**Conclusion:**

Wrist dorsiflexion/palmar flexion can affect median nerve deviation and cross-sectional area in patients with carpal tunnel syndrome. High-frequency ultrasound is helpful to detect such an effect and can also help determine the severity of carpal tunnel syndrome, which is worthy of clinical promotion.

## 1. Introduction

Carpal tunnel syndrome is one of the most common focal compression mononeuropathy [1], which is caused by the stenosis of the bone duct and the chronic inflammatory changes of soft tissue in patients over a long period of time, leading to the thickening of ligaments, thickening of tendons and muscles, and nerve edema. As a result, the median nerve, the nerve in charge of finger sensation, is squeezed in the carpal tunnel, causing motor, sensory, and autonomic nerve dysfunction. The pathological basis is that the median nerve is stuck in the carpal tunnel at the wrist. The surface of the carpal tunnel is bounded by the transverse carpal ligament, and the lateral and inferior aspects are bounded by the carpal bone and its fibrous covering and the interosseous ligament. Because of extrinsic compression, smaller lumen itself, and increased volume and number of luminal contents, the median nerve is vulnerable to injury, leading to recognized causes of work disability [2]. Radial carpal tunnel syndrome is mainly for the palm side and the radial side of the three-and-a-half paresthesia, which can seriously appear with symptoms such as hand muscle atrophy and weakness [3], can appear with positive median nerve compression tests, and may cause numbness in the fingers, palms, and wrist, tingling, pain, stiffness, or a host of other feel anomalies. Severe pain will even involve the entire upper limbs (elbow, shoulder), affecting work and life. Neurophysiological examination is the main standard used to diagnose carpal tunnel syndrome in clinical practice, but there are many limitations such as many affected factors, inability to visually observe the internal structure of the carpal tunnel, and inability to identify internal morphological changes [4]. High-frequency ultrasound has the advantages of low cost, short time, and good patient tolerance. It has been used in carpal tunnel syndrome in recent years and can help diagnose abnormalities in the carpal tunnel structure [5]. Activities such as wrist dorsiflexion/palmar flexion have an important impact on the median nerve in patients with carpal tunnel syndrome [6]; however, there are still few studies to evaluate wrist movement by high-frequency ultrasound for median nerve deviation and cross-sectional area changes. Therefore, in this study, we observed the position deviation and cross-sectional area changes of the median nerve during wrist dorsiflexion/palmar flexion in patients with carpal tunnel syndrome by high-frequency ultrasound to investigate the diagnostic value of high-frequency ultrasound and its significance in wrist movement.

## 2. Methods

### 2.1. Patients

From November 2019 to December 2021, 85 patients who presented to our department and were diagnosed with carpal tunnel syndrome were collected, with a total of 110 affected wrists. There were 20 males and 90 females with a mean age of 50 ± 8 years. Inclusion criteria were as follows: (1) abnormal sensation of three-and-a-half fingers on the radial side, atrophy and weakness of hand muscles, and limited thumb opposition function; (2) positive Tinel sign, and/or positive Phalen test, and/or positive median nerve compression test. A positive Tinel's sign was defined as percussion from the forearm distally along the course of the median nerve and numbness discomfort in the median innervated area during percussion in the carpal tunnel area. A positive Phalen test was defined as having the patient's wrist held in maximal flexion and experiencing numbness discomfort in three fingers on the radial side within 60 seconds. A positive median nerve compression test was defined as the presence of numbness discomfort in the skin of the median nerve innervated area within 30 seconds when the examiner compressed the carpal tunnel site with the thumb; (3) abnormal neurophysiological tests; and (4) stable general health, carpal tunnel syndrome symptoms within 3 months. Exclusion criteria include previous history of trauma, combined rheumatoid arthritis and liver and kidney dysfunction and dysfunction of other vital organs, tumors or bleeding, and coagulation diseases. All patients were informed and signed a consent form. The study protocol was approved by the Ethics Committee of our hospital.

### 2.2. Severity Grade

According to Stevens' criteria, 110 affected wrists were divided into the mild group (38 sides), the moderate group (30 sides), and the severe group (42 sides). Twenty-five healthy controls with 50 carpal canals were also selected. All of them were healthy subjects with normal upper limb development (male: two-finger pinch force of 177 inch-lbs, three-finger pinch force of 210 inch-lbs, grip force of 376 inch-lbs, wrist flexion force of 437 inch-lbs, and wrist extension force of 352 inch-lbs; female: two-finger pinch force of 127 inch-lbs, three-finger pinch force of 148 inch-lbs, grip force of 226 inch-lbs, wrist flexion force of 232 inch-lbs, and wrist extension force of 198 inch-lbs); left and right sides are basically symmetric.

### 2.3. Method

#### 2.3.1. High-Frequency Ultrasound

Philips IU22 and ALOKAProsounda10 color Doppler ultrasound diagnostic apparatus with linear array probe were used for measurement. All patients and healthy volunteers underwent high-frequency ultrasound examinations. In the longitudinal section of the nerve, it showed a fascicular structure with multiple low gyrus vocal cords (nerve fascicles) arranged in parallel and spaced by linear hyperechoic phases (nerve fascicles). In the cross-section, it shows a cribriform structure, the hypoechoic nerve bundle is round, and the nerve trunk is surrounded by a hyperechoic epineurium. The scanning plane of the ultrasound probe was parallel to the longitudinal axis of the palm, and the position, direction, and cross-sectional area of the median nerve were measured and recorded. Three measurements each were taken and averaged.

#### 2.3.2. Neurophysiological Testing

All patients with carpal tunnel syndrome underwent neurophysiological testing. Electromyography (model: Dantec KeyPoint, Denmark) was used for measurement in patients with carpal tunnel syndrome in the neck of the contralateral side bending, the shoulder blade sinking, shoulder joint outreach, shoulder joint extorsion, elbow joint, forearm supination, wrist extension after stretch, each finger joint stretching (especially the thumb and forefinger, middle finger, and ring finger), and position of the median nerve sensory conduction velocity, feeling the incubation period of time and moving point fluctuation. Using the forward method, the thumb and middle finger innervated by sensory fibers of the median nerve were stimulated with bipolar stimulation, and surface electrodes were recorded about 1 cm above the transverse wrist striae to record sensory conduction velocity, sensory latency time, and sensorimotor point fluctuation amplitude, respectively.

### 2.4. Statistical Analysis

Continuous variables were presented as the mean ± standard deviation, and the deviation of the median nerve and changes in cross-sectional area during wrist dorsiflexion/palmar flexion were compared using a *t*-test. The location and cross-sectional area of the median nerve were compared between the carpal tunnel syndrome groups of different severity and the control group using a *t*-test. Categorical variables were presented as frequencies (percentages). Spearman correlation was used to analyze the correlation between median nerve location and cross-sectional area and neurophysiological parameters in patients with carpal tunnel syndrome. Two-sided *P* < 0.05 was considered statistically significant. Data were analyzed using SPSS statistics 21.0 (IBM SPSS, Armonk, NY).

## 3. Results

### 3.1. The Clinical Characteristics of Patients with Carpal Tunnel Syndrome Are Shown in Table 1

A total of 85 patients and 110 affected wrists were included in this study. The mean age of the patients was 50 ± 8 years, the proportion of males was 18%, and the disease duration was 2.3 ± 1.2 years. Of the 105 affected wrists, 53.6% were positive for Tinel's sign, 80.9% were positive for Phalen's test, and 85.5% were positive for the median nerve compression test. In terms of neurophysiological parameters, sensory latency time was 5.12 ± 0.53 ms, and sensory conduction velocity was 32.12 ± 3.44 m/s. In terms of severity grading, 38 patients (34.5%) had mild carpal tunnel syndrome, 30 patients (27.3%) had moderate carpal tunnel syndrome, and 42 patients (38.2%) had severe carpal tunnel syndrome.

### 3.2. Deviation and Cross-Sectional Area of the Median Nerve during Wrist Dorsiflexion/Palmar Flexion in Both Groups

As shown in Table 2, the distance between the proximal median nerve and the transverse carpal ligament, the distance between the distal median nerve and the transverse carpal ligament, and the cross-sectional area were decreased in the carpal tunnel syndrome group and the control group during wrist palmar flexion compared with wrist dorsiflexion. When the wrist movement pattern was changed in the carpal tunnel syndrome group, the mean decrease in the proximal distance offset of the median nerve was 0.03 ± 0.01 mm, which was significantly lower than 0.07 ± 0.01 mm in the control group, and the difference was statistically significant (*P* < 0.01); when the wrist movement pattern was changed in the carpal tunnel syndrome group, the mean decrease in the distal distance offset of the median nerve was 0.03 ± 0.01 mm, which was significantly lower than 0.07 ± 0.02 mm in the control group, and the difference was statistically significant (*P* < 0.01); and when the wrist movement pattern was changed in the carpal tunnel syndrome group, the mean decrease in the cross-sectional area was 0.02 ± 0.01 cm^2^, which was significantly lower than 0.04 ± 0.01 cm^2^ in the control group, and the difference was statistically significant (*P* < 0.01).

### 3.3. Location and Cross-Sectional Area of Median Nerve in Carpal Tunnel Syndrome Groups of Varying Severity versus Controls

As shown in Table 3, there were significant differences in the vertical distance and cross-sectional area of the median nerve from the transverse carpal ligament at the proximal and distal ends in patients in the mild, moderate, and severe groups compared with the control group (*P* < 0.05). Compared with the mild group, there were significant differences in the vertical distance and cross-sectional area of the median nerve at the proximal end in the moderate group (*P* < 0.05). Compared with the mild group, there were significant differences in the vertical distance and cross-sectional area of the median nerve between the proximal and distal ends in the severe group (*P* < 0.05). Compared with the moderate group, there were significant differences in the vertical distance and cross-sectional area of the median nerve between the proximal and distal ends in the severe group (*P* < 0.05).

### 3.4. Correlation Coefficients between Median Nerve Location and Cross-Sectional Area in the Carpal Tunnel and Neurophysiological Parameters in Patients with Carpal Tunnel Syndrome

As shown in Table 4, in the neurophysiological examination of patients with carpal tunnel syndrome, the proximal vertical distance of the median nerve was correlated with the detection parameters, positively correlated with sensory latency (*P* < 0.05), and negatively correlated with sensory conduction velocity (*P* < 0.05). The vertical distance of the distal end of the median nerve was also correlated with the measured parameters, which was significantly positively correlated with sensory latency (*P* < 0.05) and significantly negatively correlated with sensory conduction velocity (*P* < 0.05).

## 4. Discussion

The carpal tunnel joint is composed of flexor support band and carpal sulcus. The superficial and deep flexor tendons of fingers and common tendon sheath of flexor muscle, flexor pollicis longus tendon, and its tendon sheath and median nerve are in the canal. The carpal bones that make up the wrist form an arch, projecting at the back of the hand and receding at the palm. The groove on the palm side, called the carpal groove, is covered by a tough connective tissue sheath flexor retinaculum that forms a bony fibrous tube, the carpal tunnel. In this study, we found that the distance between the proximal end of the median nerve, the distance between the distal end of the median nerve, and the cross-sectional area were significantly lower during the palmar flexion of the wrist in patients with carpal tunnel syndrome compared with those during wrist dorsiflexion. Compared with the control group, there were significant differences in the distance and cross-sectional area between the proximal and distal ends of the median nerve in patients in the mild, moderate, and severe groups. Notably, the distance between the proximal and distal ends of the median nerve in patients with carpal tunnel syndrome had a correlation with nerve detection parameters, a significant positive correlation with sensory latency, and a significant negative correlation with sensory conduction velocity.

Carpal tunnel syndrome is more common in middle-aged patients, especially middle-aged women, while male patients are often accompanied by occupational history. More than 30% of patients with carpal tunnel syndrome have bilateral symptoms of median nerve injury [7]. At present, the diagnosis of carpal tunnel syndrome basically identified by symptoms and signs combined with nerve physiology check can be used to check the neurons, peripheral nerve, and nerve muscle joint and muscle itself and the function of the state, which helps more to the diagnosis of neuromuscular disorders but cannot identify neurophysiology examination of carpal tunnel [8] neural structure characteristics and morphological changes in positioning which is not clear. In addition to the advantages of safety and noninvasiveness, short detection time, and low cost, high-frequency ultrasound can be used to assess parameters such as the size, blood flow, and mobility of the cross-sectional area of the median nerve [9]. In addition, high-frequency ultrasound can also provide anatomical variations and morphological changes of the median nerve, which helps to identify the factors causing carpal tunnel syndrome [10].

Studies have shown that the cross-sectional area of patients with carpal tunnel syndrome is significantly increased, which is the best ultrasound index for the diagnosis of carpal tunnel syndrome, and most cross-sectional area studies are measured at the carpal tunnel inlet, that is, the pisiform bone level [11]. This is consistent with the measurement method in this study. At present, there are few reports on the position deviation and cross-sectional area of the median nerve in the carpal tunnel during wrist movement in patients with carpal tunnel syndrome at home and abroad. In this study, we found that wrist motion had an effect on the cross-sectional area change of the median nerve at the pisiform bone level, and this effect was significantly smaller in patients with carpal tunnel syndrome than in healthy controls. In addition, we found that wrist movement also affected the median nerve position shift, and in patients with carpal tunnel syndrome, such position shift was also significantly reduced. This may be because carpal tunnel syndrome is often accompanied by chronic inflammatory hyperplasia of the synovium of the transverse carpal ligament and tendons, which can adhere to the perineurium, resulting in reduced movement and morphological changes of the median nerve [12].

This study found that compared with the control group, there were significant differences in the distance and cross-sectional area between the proximal and distal ends of the median nerve in the mild, moderate, and severe groups. This also indicates that high-frequency ultrasound is helpful for grading the severity of carpal tunnel syndrome, which may help us to choose subsequent treatment options [13]. For patients with severe carpal tunnel syndrome, surgical treatment is recommended as the first choice [14]. In patients with carpal tunnel syndrome, median nerve injury may occur in the early stage, mainly manifested as prolonged sensory latency and slow sensory conduction velocity [15]. In this study, we analyzed the correlation between the location and cross-sectional area of the median nerve and electrophysiological parameters and found that the proximal distance and distal distance of the median nerve at the level of the pisiform bone were positively correlated with sensory latency and negatively correlated with sensory conduction velocity, which indicated that high-frequency ultrasound could be helpful for early detection of neuropathy in patients [16].

In summary, wrist dorsiflexion/palmar flexion can have an impact on median nerve excursion and cross-sectional area in patients with carpal tunnel syndrome. High-frequency ultrasound helps to detect such effects and also helps to determine the severity of carpal tunnel syndrome.

## Figures and Tables

**Table 1:** Clinical characteristics of patients with carpal tunnel syndrome.

	Carpal tunnel syndrome
Number of affected wrists, *n*	110
Age (year)	50 ± 8
Male ratio, *n* (%)	20 (18)
Course of the disease	2.3 ± 1.2
Tinel sign positive, *n* (%)	59 (53.6)
Phalen test positive, *n* (%)	89 (80.9)
Median nerve compression test positive, *n* (%)	94 (85.5)
Sensory latency (ms)	5.12 ± 0.53
Sensory conduction velocity (m/s)	32.12 ± 3.44
Grade of severity	
Mild	38 (34.5)
Moderate	30 (27.3)
Severe	42 (38.2)

**Table 2:** Deviation and cross-sectional area of median nerve during wrist dorsiflexion/palmar flexion in carpal tunnel syndrome group and control group.

	Carpal tunnel syndrome group			Control group		
	Dorsiflexion	Palmar flexion	Offset/change in cross-sectional area	Dorsiflexion	Palmar flexion	Offset/change in cross-sectional area
Distance between the proximal normal middle nerve and the transverse carpal ligament (mm)	2.58 ± 0.40	2.55 ± 0.39	0.03 ± 0.01	3.01 ± 0.38	2.94 ± 0.38	0.07 ± 0.01^∗^
Distance between the distal normal middle nerve and the transverse carpal ligament (mm)	2.13 ± 0.36	2.10 ± 0.36	0.03 ± 0.01	2.46 ± 0.37	2.39 ± 0.37	0.07 ± 0.02^&^
Cross-sectional area (cm^2^)	0.18 ± 0.06	0.16 ± 0.06	0.02 ± 0.01	0.09 ± 0.04	0.05 ± 0.03	0.04 ± 0.01^#^

^∗^The proximal distance of the median nerve was significantly less shifted during dorsiflexion/palmar flexion in the carpal tunnel syndrome group compared with the control group, *P* < 0.01. ^&^Distal end distance deviation of median nerve during dorsiflexion/palmar flexion was significantly smaller in carpal tunnel syndrome group compared with control group, *P* < 0.01. ^#^Compared with the control group, the cross-sectional area of the median nerve was significantly smaller in the carpal tunnel syndrome group during dorsiflexion/palmar flexion, *P* < 0.01.

**Table 3:** Location and cross-sectional area of median nerve in carpal tunnel syndrome group and control group with different severity.

	Mild group	Moderate group	Severe group	Control group
Distance between the proximal normal middle nerve and the transverse carpal ligament (mm)	2.77 ± 0.36^∗^	2.56 ± 0.40^∗^&	2.38 ± 0.34^∗^&#	2.96 ± 0.38
Distance between the distal normal middle nerve and the transverse carpal ligament (mm)	2.21 ± 0.32^∗^	2.18 ± 0.40^∗^	1.97 ± 0.34^∗^&#	2.41 ± 0.37
Cross-sectional area (cm^2^)	0.13 ± 0.04^∗^	0.16 ± 0.04^∗^&	0.21 ± 0.05^∗^&#	0.07 ± 0.03

^∗^Compared with the control group, *P* < 0.05; ^&^compared with mild group, *P* < 0.05; ^#^compared with the moderate group, *P* < 0.05.

**Table 4:** Correlation coefficients between median nerve location and cross-sectional area and electrophysiological parameters in the carpal tunnel in patients with carpal tunnel syndrome.

	Vertical distance between median nerve and transverse carpal ligament		Cross-sectional area
	Near side	The distal end	
Sensory latency (ms)	0.468^∗^	0.430^∗^	-0.012
Sensory conduction velocity (m/s)	-0.449^∗^	-0.449^∗^	0.155

^∗^Spearman correlation analysis, *P* < 0.05.

## Data Availability

The data used to support the findings of this study are available from the corresponding author upon request.
